# Object-Oriented Technology Model of Regional Industrial Economic Innovation Project Management System

**DOI:** 10.1155/2022/4118699

**Published:** 2022-08-09

**Authors:** Weiwei Zhang

**Affiliations:** Shengda Trade Economics & Management College of Zhengzhou, Zhengzhou 451191, China

## Abstract

Managers have a deeper understanding of computer technology, network technology, and communication technology, which is also a necessary condition for the implementation of project management information. It plays an important role in improving the performance of regional resource-based industry and high-tech service industry. By analyzing the current situation of the company's project management, the project management and management processes are standardized and the management of project quality, progress, contract, and cost through the design system is completed, so that the various resources of the project can be effectively and rationally allocated and utilized. Information communication inside and outside the project is more convenient, smooth, and fast, and more standardized operating procedures can be carried out. This paper also improves the level of local government governance, shapes the cultural connotation of innovation, openness, and cooperation, and strengthens the cultivation and flow of social elements. A series of policy suggestions are put forward in building the capacity system of both sides of industrial integration, thus greatly improving the overall project management level and the company's decision-making and analysis ability, so as to achieve fine and precise management objectives.

## 1. Introduction

Project management is a behavior that runs through the project life cycle. The so-called project management is the project manager, under the constraints of limited resources, using the systematic views, methods, and theories, to effectively manage all the work involved in the project. That is, to plan, organize, command, coordinate, control, and evaluate from the beginning of the project investment decision to the end of the project, so as to achieve the goals of the project. Project management is characterized by specificity, universality, innovation, and temporariness [1].

How to manage a project? We must first define the needs of the project, during the project planning and project execution phases, address and meet the needs, concerns, and expectations of stakeholders, and balance project factors, including scope, quality, schedule, budget, and risk, which compete with each other, i.e., mutual restraint. A change in any one of these factors will affect at least one other factor. For projects to progress smoothly and successfully, companies must be able to properly analyze project status and balance project requirements. When the project management organization is at a mature stage, the scope and governance space of project management will also become broader, and we will refine it into program management and portfolio management. They have different management and operation modes. Portfolio management refers to the selection and support of multiple projects or project investments under the guidance of available resources and enterprise strategic plans. Project portfolio management is to ensure that the project meets the strategic goals of the enterprise through project evaluation and selection and multiproject portfolio optimization, so as to maximize the enterprise income. We must conduct targeted management according to the characteristics of the project to improve the efficiency and quality of project management and be consistent with the strategy of the organization, forming a set of standardized organization-level project management processes [2].

In operation, enterprises achieve commercial benefits or business goals by combining various resources, skills, technologies, and concepts of projects, and good project management is directly related to the economic benefits of enterprises. This is achieved in accordance with the project quality required by the user. The success of the project is inseparable from the internal support of the enterprise. The internal management mechanism and process, the rational allocation of resources, the implementation of project experience, and the identification and response of project risks are all valuable experiences of the project. However, for the senior managers of enterprises and institutions, the huge organizational structure and the increasing number of projects all affect the senior managers' in-depth understanding of the project and the progress tracking. In this case, it is very easy for project management problems to spiral out of control. Therefore, it is necessary for enterprise executives to establish a set of project management organizational structure and processes to ensure the overall control of the project so that the project objectives can be successfully achieved [3]. The object-oriented economic innovation project management mechanism is shown in Figure 1, based on the object-oriented characteristics.

This study will combine the current situation of the company's project management, standardize the project management and management process, using the coupling evaluation model, the integration of resource industry, and high-tech service industry, through the project quality, progress, contract, and cost management, improve the company's decision analysis ability, strengthen the project performance management ability, improve the project management level, and realize the refined and precise management objectives [4].

## 2. State of the Art

So far, project management has become not only a management behavior but also an important management discipline, a leading scientific management skill that guides the construction of the entire project management industry [5].

At present, a complete set of project management knowledge system guidelines has been formed in the field of project management, namely, the PMBOK® Guide, which is a set of recognized professional standards for project management. Because the guide is of certain importance and practicality, and its certification system is also very rigorous and scientific, so it is applicable to the management guidance of most projects. PMBOK also serves as a global management standard [6]. In PMBOK, the five stages of initiation, planning, execution, monitoring, and closing constitute the complete project management process, and the project management discipline is also divided into 9 knowledge areas: overall project management, project scope management, project time management, project cost management, project quality management, project human resource management, project communication management, project risk management, and project procurement management [7].

Domestic organizational-level project management is mainly concentrated in the fields of telecommunications, IT, R&D, manufacturing, and real estate. Among them, Huawei, as a leader in the communication industry, the famous IPD process is the essence of its implementation project management. The IPD process, which is integrated product development, is a set of product development models, concepts, and methods. At that time, CMM was not mature enough as a project management system. During the project implementation process, Huawei gradually implemented it according to Ren Zhengfei's famous three-step principle, namely, “first rigidity, then solidification, and then optimization,” and finally formed a complete set of its own. The software development system is called IPD. In the real estate industry, Vanke began to implement organizational-level project management methods in the early stage. Now, Vanke's organizational-level project management has developed to a higher level than that of the same industry. In the process of project management practice, organizational-level project management has become an important feature that distinguishes Vanke from other real estate companies [8].

In terms of input of resources, capital, labor, and technology, ethnic areas only have the advantage of resource endowment, and the selection and cultivation of advantageous industries is the strategic direction for ethnic areas to achieve leapfrog growth. The long history of industrial development and evolution in ethnic areas has gradually created an industrial layout with the energy industry, mining industry, agriculture, tourism, and other industries as pillars [9]. Among them, resource-based industries have made great contributions to the economic development of ethnic areas and are highly relevant. At present, it is facing a major industrial development dilemma and other practical problems. It includes low industrial level, insufficient scientific and technological innovation ability, imperfect supporting service system, and large external environmental constraints, which has attracted the attention of many scholars. When Zhou Minliang reflected on the economic development mode of ethnic areas, he first affirmed that the economic development of ethnic areas should be based on the regional foundation, with resource development and industrial upgrading as the main line, but at the same time he also pointed out that there is a “resource-dependent economy and industrial structure optimization and upgrading in ethnic areas.” “Contradiction between sustainable development and resource development, environmental protection” and looking at the existing research on resource-based industries in ethnic areas, we can basically summarize three research lines based on the above two contradictions [10]. One is the problem of industrial structure in ethnic areas, most of which involve resource-based industries, and the other is the development of resource-based industries and resources in ethnic areas, the relationship between the environment, and the third is the innovation and transformation of resource-based industries in ethnic areas [11].

## 3. Methodology

### 3.1. Construction and Measurement of the Evaluation Index System for the Integration of Regional Industry and High-Tech Service Industry

In this study, the evaluation of the integration of resource-based industries and high-tech service industries is carried out using a coupled evaluation model. The model consists of two major industrial subsystems, namely, resource-based industries and high-tech service industries, and specific evaluation indicators are selected for each subsystem [12]. The existing literature studies the integration of the equipment manufacturing industry and the high-tech service industry. On the one hand, the definition of the high-tech service industry is basically the same as this research. On the other hand, the equipment manufacturing industry has the attribute of heavy industry [13]. According to this attribute, this research is believed that resource-based industries can also be used for reference. Therefore, this document is mainly used to describe the development and changes of the two industries from four aspects: industrial development scale, industrial growth level, industrial opening level, production efficiency and benefit and establish an industrial integration level evaluation System. Among them, the scale of industrial development mainly reflects the basis of the integration of the two industries. They are in a specific industrial field, and they are linked together to form a regional industry because of their commonality and complementarity. When there are a certain number of enterprises, personnel, and industrial output value in the region, it means that the two industries have developed to a certain stage, and at this time, various industries may appear in the industry. Problems can only be solved by interindustry cooperation [14]. At this time, the demand for industrial integration begins to emerge; the level of industrial openness reflects the path and possibility of the integration of the two industries. The more open the two industries are, the more conducive to personnel exchanges and business interaction between the two. The opening is a necessary way for industrial integration; industrial growth strength, and production efficiency, and benefits represent the potential for deep integration of the two industries. On the one hand, the growth strength of the industry provides both parties with conditions for integration, including the ability to transform traditional production processes [15], high-tech R&D, and update and commercialization capabilities. On the other hand, production efficiency and benefits ensure that industrial integration can continue. Both industries focus on obtaining higher levels of economic benefits. Therefore, in the process of industrial integration, it is essential to obtain production benefits and realize the improvement of production efficiency, and the improvement of benefits will further promote the transition of industrial integration from technology and knowledge integration to industry, business, and market integration. The specific evaluation index system is shown in Table 1.

First, the power function and indicators are standardized. After distinguishing the positive and negative of the indicators included in the subsystem, the efficacy function is introduced to process the indicators, as follows:

(1) $$\begin{array}{c} \text{positive}\left(\text{effectiveness}\right)\text{indicators}:U_{ij}=\frac{\left(X_{ij}-\min X_{ij}\right)}{\left(\max X_{ij}-\min X_{ij}\right)},\\ \text{inverse}\left(\text{cost}-\text{type}\right)\text{indicators}:U_{ij}=\frac{\left(\max X_{ij}-X_{ij}\right)}{\left(\max X_{ij}-\min X_{ij}\right)}. \end{array}$$

Among them, *U*_*ij*_ is the efficacy coefficient of the index *j* of system *i*, which reflects the contribution of *X*_*ij*_ to the coupled system, and the *j*th variable value of the ith order parameter of *X*_*ij*_.

Secondly, the information entropy is used to determine the index weight.

(2) $$\begin{array}{c} \text{Calculate the index information entropy}:E_{j}=-\ln\;{\left(m\right)}^{-1}\times \sum_{i=1}^{m}\left(p_{ij}\times \;\ln\;p_{ij}\right),\\ \text{calculate the weight of each indicator:}W_{j}=\frac{\left(1-E_{j}\right)}{\left(n-\sum E_{j}\right)},\\ \text{among them},m\text{ represents the number of years of evaluation}:p_{ij}=\frac{u_{ij}}{\sum_{i=1}^{m}u_{ij}}. \end{array}$$

If *Pij*  = 0, then define *Pij* × Inpij  = 0

The weights of each index in the evaluation system calculated by the entropy method are also listed in Table 1.

Third, evaluate the comprehensive development level.

(3) $$\begin{array}{c} \text{Measured by linear weighting method}:U_{1}=\sum_{t=1}^{m}W_{j}X_{ij};U_{2}=\sum_{e=1}^{n}W_{j}Y_{ij}. \end{array}$$

Among them, *u*_1_ and *u*_2_ represent the comprehensive development index of the high-tech service industry and resource-based industry, respectively, *t* and *e* represent the number of evaluation indicators of the two subsystems, respectively, *Wj* is the indicator weight calculated previously, *Xij* are *Yij* are calculated previously The contribution degree of the *j*th index of the two subsystems in the *i*th year takes the value.

Finally, the coupling coordination degree is evaluated.

(4) $$\begin{array}{c} \text{Coupling Relevance}:C=\sqrt{\frac{U_{1}\times U_{2}}{{\left(U_{1}+U_{2}\right)}^{2}}},\\ \text{Coupling coordination degree}:D=\sqrt{C\times T}. \end{array}$$

Among them, *T*  = *αU* 1 + *βU* 2, which represents the comprehensive development level index of the two industries, *α* and *β* are undetermined coefficients.

This study argues that *U*_1_ and *U*_2_ represent the composite development index of high-tech services and resource-based industries respectively, so both *α* and *β* are valued at 0.5. The value of *D* is between [0, 1]. The larger the value, the more orderly development of the industrial system portfolio, and the more coordinated and integrated development between industries can be achieved. The specific evaluation criteria are shown in Table 2.

### 3.2. The Impact of Regional Industries on Industrial Economic Performance

The level of integration and development of resource-based industries and high-tech service industries depends on the original industrial foundation and environment in the region [16]. Through the spillover and sharing of technical information, industrial clusters promote the innovation of enterprises; through the spillover and sharing of industry and market information, as well as by enhancing trust among enterprises, reducing transaction costs, and promoting cooperation between enterprises. As a traditional industry with a long development time, resource-based industries have become stable in various regions. However, as an emerging industry, the high-tech service industry is not only mainly concentrated in the developed eastern regions but also shows a phenomenon of further agglomeration in the eastern regions. High-tech resources have a polarization effect, which may lead to two spatial effects of industrial integration [17]. One is that as high-tech resources continue to accumulate in relatively developed areas, a siphon effect is generated on adjacent backward areas, resulting in negative industrial integration. To the spillover effect, the second is the emergence of “late-mover advantages;” that is, the more a region's economy lags behind the national technology-leading region, the easier it is for the region to advance to the technological frontier through technology diffusion, and industrial integration can enhance the flow scale and scope of mobile production factors. So that the achievements of industrial integration in adjacent areas can provide support for the development of local industries so that industrial integration has a positive spillover effect [18]. The special feature of the resource-based industry is that its regional development foundation is more stable than that of the central and eastern regions, and it is an important part of the industrial structure. The well-developed industrial foundation and policies of resource-based industries in the region will help drive them to seek the results of industrial integration in neighboring regions through industrial cooperation and alliances. At the same time, due to the real dilemma of brain drain in the region, the siphoning effect may offset the technology diffusion effect. Therefore, based on the above analysis and the actual situation, the following assumptions are made:

 
*Hypothesis 3a*. The integration of resource-based industries and high-tech service industries around the region has a positive spillover effect on the economic performance improvement of local resource-based industries
 
*Hypothesis 3b*. The integration of resource-based industries and high-tech service industries around the region has a negative spillover effect on the economic performance improvement of local resource-based industries

First of all, according to the above-given analysis, the general panel regression model of the integration of regional resource-based industries and high-tech service industries on the economic performance of resource-based industries is constructed as follows:

(5) $$\begin{array}{c} Y_{i,t}=\beta_{0}+\beta_{1}{\text{Conv}}_{i,t}+\sum {\text{ Control }}_{i,t}+\varepsilon_{i,t}. \end{array}$$

Among them, *i* represents the individual, *t* = 1,2,…, T represents the sample research time, *Yi*, *t* represents the economic performance of resource-based industries, Convi, *t* represents the level of industrial integration, Controli, *t* represents all control variables, *εi*, *t* is a random disturbance term.

(6) $$\begin{array}{c} Y_{i,t}=C+\beta_{1}{\text{Conv}}_{i,t}+\beta_{2}{\mathrm{Gov}}_{i,t}+\beta_{3}{\text{Conv}}_{i,t}\times {\mathrm{Gov}}_{i,t}+\sum {\mathrm{Control}}_{i,t}+\varepsilon_{i,t}. \end{array}$$

Among them, *Govi*, *t* represent the adjustment variables of the government governance model, and the variables of social elements and relational cultural elements are also introduced according to this model. For the specific variable symbols, please refer to the variable definition table.

At the same time, a corresponding spatial econometric model is constructed to further investigate the spatial spillover effect of the economic performance of industrial integration [19]. At present, the widely used spatial econometric models include the spatial lag model (SLM), the spatial error model (SEM), and the spatial Durbin model (SDM). It is also affected by independent variables in adjacent regions, which can more accurately identify the key factors affecting the dependent variable, and better capture the spatial correlation of the dependent variable and the spatial spillover effect of the independent variable. According to Elhorst's point of view, generally, the spatial Durbin model can be selected as a general model for construction, and then the LM test, Wald test, and LR test can be used to judge whether it can be simplified into a spatial lag model and a spatial error model, and the following spatial econometric model can be constructed:

(7) $$\begin{array}{c} Y_{i,t}=\alpha_{i}+\rho \sum_{j=1}^{N}W_{i,j}Y_{j,t}+\beta X_{i,t}+\varphi \sum_{j=1}^{N}W_{j,t}X_{j,t}+u_{i},\\ u_{i}=\lambda W\mu_{i}+\varepsilon_{i}. \end{array}$$

Among them, *Yi* are *t* are dependent variables, representing the economic performance of regional resource-based industries; *X* represent core explanatory variables and a series of control variables; *i* and *j* represent different provinces, and *t* represent different years; *ρ* and *λ* represent spatial autocorrelation regression coefficients. If *ρ* ≠ 0 and *φ*  = 0, the model is a spatial lag model, explaining the influence of the explained variables in the neighboring provinces on the explained variables in the region; if *λ* ≠ 0 and *ρ*  = 0, the model is a spatial error model, inversely. It reflects the influence of other unconsidered factors other than explanatory variables in neighboring provinces on the explained variables in the region; if *ρ* ≠ 0, *φ* ≠ 0, and *λ*  = 0, the model is a spatial Durbin model, which not only considers neighboring provinces In addition, the influence of other explanatory variables and control variables included in the model in neighboring provinces on the explanatory variables in this region is also considered.

### 3.3. The Impact of Regional Industries on Industrial Economic Performance

Industrial economy is an important component of economic development, and from the refinement of the industrial economy to distinction, the industry can be based on the nature of consumer processing and the use of its products to implement industrial distribution, can also implement industrial classification, therefore, from the industrial internal and local work to distinguish, the industrial economy can be divided into various industries. The integration of regional high-tech service industry and traditional industries can not only make the original independent technical models and technical capabilities of the industries have a common platform foundation but also introduce external specialized knowledge capital and innovation achievements into the innovation and R&D process of traditional industries and help traditional industries to achieve innovation. The allocation of R&D resources in a wider range can also improve the environmental momentum of innovation and R&D in traditional industries through the sharing of technology and knowledge, explore new interfaces for industrial integration, and promote the formation of cross-border models of innovation and R&D activities in traditional industries and improve the efficiency of innovation and R&D. However, there are also different opinions in academia [20]. For example, “Solo's paradox” and “Gordon's doubt” believe that the development of information technology may not bring about productivity improvement, and some scholars have proposed that the impact of new technologies on the innovation efficiency of traditional industries is irrelevant or adverse effects, such as Shishang and other representative industries of the high-tech service industry, information and communication industry, and technology service industry, although the radiation area is large, due to insufficient connection depth and insufficient radiation intensity, the improvement of innovation efficiency has not yet been formed in an effective way. Although regional resource-based industries have undergone several rounds of adjustments such as supply-side reforms, the problem of overcapacity has not been fundamentally changed, and the contradiction between oversupply and demand cannot be completely resolved in the short term. Many enterprises are in a state of meager profits or even losses, resulting in a lack of innovation and R&D investment capacity and intrinsic motivation. In addition, as the supply-side reform has been basically completed, the resource-based industry as a supplier of raw materials has experienced a rebound in prices. Many resource-based enterprises in the region, stimulated by short-term speculation and price increase expectations, have accumulated in the industry's “cold winter” period. The desire for innovation has been shelved again. Therefore, the current integration of resource-based industries and high-tech service industries in the region may not have a significant impact on the improvement of innovation and R&D efficiency in resource-based industries. It may even be due to the gap between the original technology models of the two parties, related talents, and funds. There are negative effects due to the lack of strength. Based on this, this study proposes the following hypotheses:

 
*Hypothesis 1a*. The integration of regional resource-based industries and high-tech service industries has a positive impact on the improvement of innovative R&D performance in resource-based industries;
 
*Hypothesis 1b*. The integration of regional resource-based industries and high-tech service industries has a negative impact on the improvement of innovative R&D performance in resource-based industries.

This study divides the innovation value chain into the innovation R&D stage from innovation input to innovation R&D output and the innovation transformation stage from the transformation of innovative R&D results to market revenue, as shown in Figure 1. The selection of indicators is based on the existing literature. Innovation R&D efficiency (IE1) mainly reflects the level and ability to convert innovation resource input into knowledge achievements. In the calculation, R&D expenditure and R&D personnel are selected as inputs, and the number of patent applications and total intangible assets are selected as intermediate outputs; innovation transformation efficiency (IE2) reflects the level of converting knowledge input and economic input into economic output. In addition to the intermediate output in the first stage, noninnovative production expenses are also selected as input variables, specifically operating costs and deductions for R&D personnel. The total number of employees, operating income, and net profit are denoted as the final output of this stage. All indicators are standardized by the “extreme value method” to eliminate the influence of negative and zero values as shown in Figure 2.

Finally, according to the calculation results, the average efficiency value is obtained by sorting out the two-stage innovation efficiency values of regional, nonregional, and national resource-based listed companies, as shown in Table 3.

At the same time, in order to show the changing trend of innovation efficiency in the two stages of regional and nonregional as shown in Figure 3.

From the comparison between regions and nonregions, the overall trend of innovation efficiency at each stage in the two regions is basically the same, but there are big differences in R&D efficiency. Except in 2014, the R&D efficiency of the region was comparable to that of the nonregional region. In other years, the R&D efficiency of the region was significantly lower than that of the nonregional region. Moreover, the regional R&D efficiency only fluctuated in a relatively low range, and the fluctuation range was small, reflecting to a certain extent. Problems such as the lack of innovative talents and poor social environment in the region make it difficult to improve the efficiency of innovation and R&D. In terms of transformation efficiency, although regions are not as good as nonregions in most years, the gap is relatively small, reflecting that the innovation transformation of resource-based industries is highly linked to industrial economic performance, and regions with higher development levels of resource-based industries have not appeared significantly. In addition, the impact of external economic environment shocks is the same as that of nonregions. In 2016, the efficiency of innovation and transformation has declined, while the impact of regional special factors is relatively low.

## 4. Result Analysis and Discussion

### 4.1. Evaluation of the Integration Level of Regional Industry and High-Tech Service Industry

Regional resource-based industries are large-scale. At present, the number of resource-based enterprises in the overall industrial enterprises above the designated size in the region accounts for about half, and in terms of total assets and employees, the proportion of resource-based enterprises is even far more than half.

Figure 4 reflects the development trend of the scale of resource-based industries in the past ten years. In 2013, the number of resource-based enterprises, fixed assets, and employees all reached the peak. Since then, all the three have fluctuated somewhat, but the maximum value did not exceed 2013.

The economic contribution rate of regional resource-based industries declined. The proportion of resource-based industries in the overall industrial development of the region reflects its contribution to the regional economic development. The overall industrial development level mainly refers to the industrial sales output value of industrial enterprises above the designated size at the price of the current year. The specific formula is: regional resource-based industries. Industry contribution rate = (regional resource-based industry sales output value/regional industrial sales output value in the current year) × 100%. From 2007 to 2016, the economic contribution rate of regional resource-based industries basically exceeded 60%.

Compared with the national average economic contribution rate of resource-based industries (Figure 5), the economic contribution rate of regional resource-based industries far exceeds the national average. However, since 2014, due to the country's vigorous promotion of supply-side reforms and changes in supply methods and structures, a number of low-end supplies have been banned, and the contribution rate of regional resource-based industries has dropped significantly, and the rate of decline is faster than the national average.

Figure 6 shows the integrated development of regional resource-based industries and high-tech service industries in the past 10 years. First of all, the overall level of regional industrial integration is between 0.3 and 0.6, that is, the transition from mild dissonance, on the verge of dissonance to reluctance to coordinate, and secondly, from the perspective of development trend, it has mainly started to show a stable growth trend after 2012. Among all regions, Qinghai and Ningxia show a high degree of integration and coordination, which is likely to be related to the local industrial structure. Therefore, compared with other regions, a certain service industry foundation is conducive to the integration and penetration of industries, and the integration and coordination of resource-based industries and high-tech service industries is also higher.

Compared with the average degree of industrial integration in other nonregional regions in China, it can be found that the overall industrial integration coordination degree of regions at the regional level was 0.493 in 2016, ranking in the middle reaches of the country and lower than that of the eastern and central regions. The degree of regional industrial integration and coordination is slightly higher than that of the West African region (including Sichuan, Chongqing, Gansu, and Shaanxi), but the difference is not obvious. In addition, the coordination degree of regional industrial integration is higher than that of the Northeast region. The main reason for the lower degree of industrial integration coordination in the Northeast region is that the integration level of Liaoning Province is not high. This is likely to be related to the local industrial layout dominated by heavy industry. Especially in Liaoning Province, the situation is still difficult to return.

### 4.2. Empirical Analysis of the Impact of Regional Industries on Industrial Economic Performance

According to the above-given variable definitions and data sorting, a total of 70 observation data in 10 years in 7 provinces (excluding Tibet) are obtained. The descriptive statistics are shown in Table 4.

First, the Ordinary Least Squares (OLSs) method was used for estimation, and the core explanatory variables and control variables were substituted into the formula. The results are shown in Table 5. The results show that the estimated coefficient of the fusion variable of regional resource-based industries and high-tech service industries is positive and significant at the 5% level. At the same time, judging from the comparison results of OLS regression, it seems to reflect that regional, nonregional, and national total samples have the effect of industrial integration on the economic performance of resource-based industries.

However, considering that the results of ordinary least squares estimation may be inaccurate, the conclusions need to be further verified. According to the results of the Hausman test, the panel fixed-effects model is selected for estimation again. Specifically, it is basically consistent with the results of the OLS regression. The industrial integration has a significant positive impact on the economic performance improvement of resource-based industries in each sample, and the regional nonregional positive impact is greater.

### 4.3. Empirical Analysis of the Impact of Regional Industries on the Innovation Performance of Resource-Based Industries

Table 6 reports the descriptive statistics of the main variables of regional resource-based enterprises. The results show that the average transformation efficiency of regional resource-based listed companies is higher than the average R&D efficiency, and the differences in R&D efficiency between enterprises are larger. The average value of the industrial integration lagging one period is 0.43, which is on the verge of dissonance, with a minimum value of 0.35 and a maximum value of 0.55. The overall value is between mild dissonance and barely coordinated. The mean value of absorptive capacity is 7.07, and the standard deviation is relatively large, indicating that the differences among listed companies in the region are very obvious.

Table 7 reports the correlation between the variables. The lag 1 period of industrial integration and innovation R&D efficiency has a significant positive impact, while it has a significant negative impact on innovation transformation efficiency; absorptive capacity and innovation efficiency at each stage have a significant positive impact. The above-given results need to be further verified by the regression model. The variance inflation factor VIF between each explanatory variable is less than 2. At the same time, in order to avoid the problem of multicollinearity, the main indicators are centralized.

This paper reports the impact of the integration of regional resource-based industries and high-tech service industries on the two-stage innovation efficiency of resource-based industries.

## 5. Conclusion

1. The regional resource-based industry is an important support for the regional economy. The overall scale of the industry occupies half of all industrial enterprises above the designated size. However, in recent years, new problems such as the decline of industrial economic contribution rate and profit rate, the threat of resource depletion, and the upgrading of environmental protection requirements have emerged. However, the technical level of regional resource-based industries is far behind the national average, and it is difficult to achieve it alone. The regional high-tech service industry has developed rapidly in recent years, and the development trend is better. Although the industrial status still needs to be improved and the service capacity needs to be improved, its penetration and integration of resource-based industries is one of the current regional industrial development trends, and it also helps to solve the problem of the insufficient technical level of resource-based industries.
2. The integration of regional resource-based industries and high-tech service industries has begun to take shape and has the economic effects of transforming the production process of resource-based industries, reducing losses, realizing business and management synergy, innovating sales models, and introducing external professional R&D services. The innovation effect and the “three wastes” monitoring and the environmental effect of ecological restoration and other good effects. However, the standardization of various related concepts, the “bridging” communication between industries and government departments, and the problem of financial pressure are all problems that affect the deepening of the integration of regional resource-based industries and high-tech service industries. At the same time, the regional talents, funds, and basic facilities are not enough compared with the developed regions in the southeast coast, which makes it difficult for high-tech R&D companies to settle in the region, but technology application companies are more likely to be introduced in the region. Therefore, the regional high-tech services are mainly platform-based service, participatory service, and infrastructure service which are the main integration modes, which are also an important direction for the further integration of regional industries in the future.
3. The level of integration between regional resource-based industries and high-tech service industries has changed from “slightly out of balance” to “barely coordinated” since 2007. It is lower than that of the eastern and central regions, and the gap has been further widened after 2013. Although the integration trend is improving, and the integration level of individual provinces is relatively high, the limited development level of the regional high-tech service industry, the poor acceptability of resource-based industries, and the weak synergy with neighboring provinces may still limit regional industries by deepening of the degree of integration.
4. The innovation R&D efficiency and innovation transformation efficiency of regional resource-based industries are both lower than those of nonregions. Among them, the gap between innovation and R&D efficiency is large, and it is more difficult for regional resource-based industries to rely solely on the industry itself to improve R&D efficiency. The integration of regional resource-based industries and high-tech service industries has a positive role in promoting innovation and R&D efficiency in a relatively long lag period, and the efficiency of innovation transformation is “first inhibited and then promoted,” indicating that regional interindustry interaction in innovation requires a certain degree of the break-in time can have a good effect. However, in nonregions, although the short-term impact of industrial integration is not significantly different from that in regions, in the long-term, the improvement of innovation performance is not as good as that in regions, which may be due to the weak innovation foundation of regional resource-based industries, which are more likely to be driven by high-tech service industries. In addition, the degree of relational education in a region has a positive moderating effect on the efficiency of industrial integration and innovation transformation, but the degree of adjustment is not high, while the efficiency of social capital allocation has a negative moderation effect on industrial integration and innovation and R&D efficiency, indicating that the limited capital tends to lean more towards less risky areas, resulting in underfunded R&D. The absorptive capacity, which is a microscopic reflection of regional social factors, has a certain positive moderating role in industrial integration and innovation and R&D efficiency, but the relationship is not stable, and the construction of regional resource-based industries absorptive capacity needs to be improved.

## Figures and Tables

**Figure 1:** Economic innovation project management mechanism of object-oriented technology.

**Figure 2:** Two-stage network model of innovation input-innovation R&D output-innovation achievement market transformation.

**Figure 3:** Trend and comparison of innovation efficiency in two stages with nonregional regions.

**Figure 4:** Development trend of regional resource-based industries.

**Figure 5:** Trend of economic contribution rate of regional resource-based industries.

**Figure 6:** Evolution of the trend of the integration development level of regional resource-based industries and high-tech service industries.

**Table 1:** Evaluation index system and weight of resource-based industry and high-tech service industry integration.

First-level indicator	Resource-based industry		High-tech service industry	
	Secondary indicators	Weights	Secondary indicators	Weights
Industrial development scale	Industrial sales output value	0.009	High-tech service industry added value	0.005
	Number of companies	0.020	Number of legal entities	0.026
	Average number of employees	0.003	Number of employees in urban units	0.007

Industry growth level	Sales growth rate	0.112	Value added growth rate	0.148
	Operating profit growth rate	0.165	Corporate unit growth rate	0.159
	Average employment growth rate	0.118	Growth rate of employees in urban units	0.123

Level of industrial openness	Fixed asset growth rate	0.183	Fixed asset investment growth rate	0.134
	Foreign capital	0.021	Foreign direct investment	0.049
	Export delivery value	0.020	Technical market transaction contract amount	0.028

Production efficiency and effectiveness	Labor productivity	0.047	Labor productivity	0.034
	Cost profit margin	0.197	Employment contribution rate	0.134
	Asset preservation and appreciation rate	0.105	Fixed asset investment effect coefficient	0.153

**Table 2:** Coordination evaluation criteria.

Coupling coordination degree (D value)	Coordination level
D ∈ (0,0.1]	Extremely out of balance
D ∈ (0.1,0.2]	Severely disordered
D ∈ (0.2,0.3]	Moderately disordered
D ∈ (0.3,0.4]	Mild disorder
D ∈ (0.4,0.5]	On the verge of dysregulation
D ∈ (0.5,0.6]	Barely coordinated
D ∈ (0.6,0.7]	Primary coordination
D ∈ (0.7,0.8]	Intermediate coordinator
D ∈ (0.8,0.9]	Well coordinated
D ∈ (0.9,1]	Quality coordination

**Table 3:** Average innovation efficiency of resource-based listed companies in main research regions from 2014 to 2017.

	Ethnic area		Non-ethnic areas		National total sample	
	R&D efficiency	Conversion efficiency	R&D efficiency	Conversion efficiency	R&D efficiency	Conversion efficiency
	Mean	Mean	Mean	Mean	Mean	Mean
2014	0.709	0.874	0.717	0.893	0.716	0.891
2015	0.642	0.798	0.679	0.818	0.674	0.816
2016	0.661	0.635	0.751	0.694	0.741	0.687
2017	0.631	0.715	0.661	0.768	0.658	0.762

**Table 4:** Descriptive statistics.

Variable	Mean	Std.	min	25% value	50% value	75% value	Max
Conv	0.42	0.05	0.29	0.38	0.43	0.45	0.56
Roe	0.12	0.08	−0.03	0.06	0.12	0.19	0.36
Pgdp	18736.86	8493.05	5264.75	13012.21	17520.51	23147.23	41255.88
Pscale	93.94	78.30	7.924	14.01	96.89	196.91	206.17
Patent	3925.76	3688.30	222	1328	2602	5846	14858
Eneff	2.64	1.68	0.77	1.51	1.86	4.55	6.21
IndusStr	0.40	0.04	0.32	0.36	0.40	0.43	0.49
Trans	0.39	0.29	0.08	0.11	0.41	0.54	1.12
Resou	1.44	0.76	0.20	0.78	1.55	2.03	3.00

**Table 5:** Ordinary least squares estimation and comparison of the economic performance impact of the integration of regional resource-based industries and high-tech service industries.

Variable	Economic performance roe (ethnic areas)	Economic performance roe (nonethnic areas)	Economic performance roe (national sample)
Conv	0.330 (1.99)	0.231 (3.53)	0.246 (4.19)
InPgdp	−0.052 (−1.43)	−0.026 (−0.61)	−0.031 (−0.78)
InPscale	0.041 (1.23)	0.080 (4.27)	0.081 (3.91)
InPatent	0.020 (1.47)	0.006 (0.48)	0.008 (0.63)
InEneff	−0.027 (−0.94)	0.030 (1.52)	0.036 (0.155)
IndusStr	−0.507 (−3.55)	−0.346 (−3.89)	−0.351 (−4.69)
InTrans	−0.063 (−1.25)	−0.066 (−1.54)	−0.087 (−2.62)
InResou	0.054 (−1.30)	0.009 (1.26)	0.012 (1.76)
_Cons	−0.372 (−1.30)	−0.537 (−1.39)	−0.531 (−1.67)
N	70	230	300
*R* ^2^	0.560	0.314	0.332

**Table 6:** Descriptive statistics.

Variable	Mean	Std.	min	25% value	50% value	75% value	Max
IE1	0.65	0.23	0.22	0.44	0.67	0.85	1.00
IE2	0.76	0.17	0.27	0.66	0.79	0.89	1.00
Conv-1	0.43	0.05	0.35	0.39	0.43	0.47	0.55
Acap	7.07	4.91	0.24	3.75	5.73	9.32	35.40
Size	2.3*e* + 06	2.9*e* + 06	1.6*e* + 05	3.3*e* + 05	1.2*e* + 06	3.0*e* + 06	1.5*e* + 07
Grow	8.95	30.60	−56.13	−7.75	6.11	27.35	158.68
Roe	1.26	10.30	−62.10	0.63	2.93	5.67	17.26
Age	17.78	2.11	12.00	16.00	18.00	19.00	23.00
Market-1	4.62	0.80	2.53	4.43	4.68	4.90	7.08

**Table 7:** Correlation analysis.

Variable	IE1	IE2	Conv-1	Aca	Size	Grow	Roe	Age	Mar-_1_
*IE* ^*1*^	1								
*IE* ^*2*^	0.314	1							
Conv-1	0.055	−0.178	1					
Acap	0.089	0.160	0.078	1			
Size	−0.627	−0.457	−0.080	−0.154	1			
Grow	−0.059	−0.047	0.251	0.044	0.018	1		
Roe	−0.009	0.136	0.126	0.086	0.004	0.307	1	
Age	−0.025	−0.110	0.266	0.080	0.024	0.063	0.061	1
Mar-1	0.136	0.112	0.385	0.111	−0.145	0.055	0.219	0.18	1

## Data Availability

The labeled data set used to support the findings of this study is available from the author upon request.
